The article "From Flies to Men: ROS and the NADPH Oxidase in Phagocytes" was published in 2021. Journal: Front Cell Dev Biol.

# From Flies to Men: ROS and the NADPH Oxidase in Phagocytes

**DOI:** 10.3389/fcell.2021.628991

**Published:** 2021-03-26

**Authors:** Zohreh Mansoori Moghadam, Philipp Henneke, Julia Kolter

**Affiliations:** ^1^Institute for Immunodeficiency, Center for Chronic Immunodeficiency (CCI), Medical Center – University of Freiburg, Faculty of Medicine, University of Freiburg, Freiburg, Germany; ^2^Faculty of Biology, University of Freiburg, Freiburg, Germany; ^3^Center for Pediatrics and Adolescent Medicine, Medical Center – University of Freiburg, Freiburg, Germany

**Keywords:** NADPH, reactive oxygen species, myeloid cells, inflammation, CGD, mitochondrial ROS, neutrophils, macrophages

## Abstract

The cellular formation of reactive oxygen species (ROS) represents an evolutionary ancient antimicrobial defense system against microorganisms. The NADPH oxidases (NOX), which are predominantly localized to endosomes, and the electron transport chain in mitochondria are the major sources of ROS. Like any powerful immunological process, ROS formation has costs, in particular collateral tissue damage of the host. Moreover, microorganisms have developed defense mechanisms against ROS, an example for an arms race between species. Thus, although NOX orthologs have been identified in organisms as diverse as plants, fruit flies, rodents, and humans, ROS functions have developed and diversified to affect a multitude of cellular properties, i.e., far beyond direct antimicrobial activity. Here, we focus on the development of NOX in phagocytic cells, where the so-called respiratory burst in phagolysosomes contributes to the elimination of ingested microorganisms. Yet, NOX participates in cellular signaling in a cell-intrinsic and -extrinsic manner, e.g., via the release of ROS into the extracellular space. Accordingly, in humans, the inherited deficiency of NOX components is characterized by infections with bacteria and fungi and a seemingly independently dysregulated inflammatory response. Since ROS have both antimicrobial and immunomodulatory properties, their tight regulation in space and time is required for an efficient and well-balanced immune response, which allows for the reestablishment of tissue homeostasis. In addition, distinct NOX homologs expressed by non-phagocytic cells and mitochondrial ROS are interlinked with phagocytic NOX functions and thus affect the overall redox state of the tissue and the cellular activity in a complex fashion. Overall, the systematic and comparative analysis of cellular ROS functions in organisms of lower complexity provides clues for understanding the contribution of ROS and ROS deficiency to human health and disease.

## Introduction

The biological system involving the formation and scavenging of reactive oxygen species (ROS) emerged more than 3 billion years ago, together with the appearance of photosynthetic organisms (Inupakutika et al., 2016). Upon discovery of ROS, their radical function was primarily considered to damage exposed cells and tissue structures. Later, it became clear that ROS are versatile in function and integral to cellular signaling in most organisms. NADPH oxidases (NOX), as major sources of ROS, play an important role in this context. Within this group, the phagocyte NADPH oxidase (NOX2) is the best-studied member. It generates large amounts of ROS in phagosomes, which function to kill ingested microbes in a direct or indirect fashion. However, homologs exist in nearly all cells of plant or animal origin (Nauseef, 2019), suggesting functions of NOX beyond the mammalian immune system.

In this review, we focus on the role of NOX and ROS signaling in professional phagocytes, where ROS have mainly been studied for their role in pathogen elimination. Yet, NOX2 can also be recruited to the plasma membrane of phagocytes leading to the generation of extracellular H_2_O_2_ (Aviello and Knaus, 2018), and NOX2-derived ROS participate in major signaling pathways, both within the individual phagocyte and surrounding cells. Additionally, mitochondria contribute substantial amounts of ROS during oxidative phosphorylation (Hamanaka and Chandel, 2010). These pathways require tight regulation, as excessive ROS produced by phagocytes may cause oxidative stress and damage in the tissues and contribute to e.g., neurodegeneration (Wu et al., 2006). A dysfunction of phagocyte NOX, on the other hand, results in chronic granulomatous disease (CGD) in humans, characterized by recurrent bacterial and fungal infections as well as granuloma formation and hyperinflammation.

Due to the different sources and potential paracrine effects, studying the effect of ROS on certain cell types and tissues is rather complex. Thus, the analysis of organisms of lower complexity can provide valuable insights. While mammals possess different types of phagocytes, i.e., granulocytes, dendritic cells, macrophages, and monocytes, the cellular immune system of insects consists only of one phagocytic cell type called hemocyte. Hemocytes can either circulate in the hemolymph or adhere to certain tissues and recognize and phagocytose foreign material, resulting in assembly of NOX and superoxide production (Browne et al., 2013). In zebrafish, on the other hand, macrophages and neutrophils can be distinguished, which share multiple characteristics with the mammalian counterparts (Linnerz and Hall, 2020). Here, we will compare ROS formation and function in phagocytes of different species and discuss the impact of phagocyte-derived ROS on cellular and tissular signaling.

## ROS Formation in Different Species

### The Evolution of NADPH Oxidase Enzymes

NOX enzymes emerged at the transition from unicellular to multicellular life (Bedard et al., 2007) and thus exist in fungi, plants, and animals. The mammalian NOX family currently contains seven members, i.e., NOX1–5 and the dual oxidases DUOX1 and 2. The enzyme evolved early in eukaryotic development. It was postulated that the ancestral type was similar to NOX1–4 (Kawahara et al., 2007). NOX1–3 and NOX4, on the other hand, emerged from a common branch, as both of these subgroups depend on the presence of p22^phox^ to be activated or stable (Kawahara et al., 2007) (Figure 1).

**FIGURE 1:** Structure and hypothetical evolution of NOX isoforms. The ancestral NOX enzyme consists of a conserved C-terminal core region including six transmembrane a-helices, two heme (Fe) groups, and a NADPH-binding cytoplasmic C-terminal domain. The conserved gp91^phox^ subunit transfers electrons from NADPH to reduce oxygen (O_2_) to superoxide anion (O_2_^−^). Later NOX isoforms acquired dependence on the activating subunit p22^phox^ or calcium. NOX1–3 and NOX4 emerged from a common branch, as both of these subgroups depend on the presence of the p22^phox^ subunit with two transmembrane a-helices. However, NOX4 solely relies on p22^phox^, while NOX1–3 require additional cytoplasmic subunits. Mammalian NOX2 additionally relies on the cytoplasmic regulators p47^phox^, p67^phox^, p40^phox^, and Rac. In contrast, NOX1 is regulated by NOXO1 and NOXA1. NOXO1 also contributes to NOX3 activation. NOX5 evolved from ancestral NOX through the acquisition of four EF hand motifs containing a Ca^2+^-binding domain, which enables activation by cytosolic calcium rather than other subunits. DUOX1/2 enzymes then emerged from NOX5 isoforms by the addition of a peroxidase domain in the N-terminal region enabling H_2_O_2_ production (Bedard et al., 2007; Kawahara et al., 2007).

The first mammalian NADPH oxidase to be discovered was NOX2, the phagocyte NADPH oxidase. The active form comprises six subunits: the integral membrane units gp91^phox^ and p22^phox^ and the regulatory subunits p40^phox^, p47^phox^, and p67^phox^ as well as the GTPase Rac, which are localized in the cytoplasm. The other NOX isoforms were discovered later and vary at the molecular level (Panday et al., 2015). In NOX1, 3, and 4, gp91^phox^ homologs form together with p22^phox^ the flavocytochrome *b*_558_, which facilitates the transfer of electrons from NADPH to reduce O_2_ to O_2_^–^. NOX1 additionally recruits Nox organizing protein 1 (NOXO1) and NOX activator 1 (NOXA1), which are homologs of p47^phox^ and p67^phox^, respectively (Panday et al., 2015). In contrast, the activation of NOX5 and DUOX1 and 2 is mediated via Ca^2+^ and does not rely on regulatory subunits.

NOX1 is widely expressed in different cell types, with particularly high expression in colonic epithelial cells (Szanto et al., 2005) and endothelial cells of the colon, and vascular smooth muscles (Hanna et al., 2004). NOX2 is predominantly expressed in phagocytes, with lower expression in vascular smooth muscle cells (Briones et al., 2011) and human endothelial cells (Buul et al., 2005). It is generally accepted to be the major ROS source in humans (Lam et al., 2010) and it is expressed in all metazoan organisms, except for nematodes and arthropodes (Sumimoto, 2008). NOX2 is the most stringently conserved NOX enzyme among vertebrates (Kawahara et al., 2007). NOX3 was detected in the inner ear of mice (Bánfi et al., 2004) and is primarily expressed in fetal tissues (Cheng et al., 2001). It is not present in frog, zebrafish, and teleost fish, which led to the conclusion that NOX3 evolved after the emergence of fish and amphibians (Kawahara et al., 2007). NOX4 is expressed in fetal tissues and the kidney (Cheng et al., 2001). It is a main NOX isoform in non-phagocytic cells, where it is located in the endoplasmic reticulum (Chen et al., 2008). Finally, NOX5 evolved from NOX1-4 through the acquisition of a Ca^2+^-binding EF hand motif, which enables activation by cytosolic calcium (Bedard et al., 2007; Kawahara et al., 2007; Touyz et al., 2019) (Figure 1). These Ca^2+^-binding motifs evolved early during evolution, as NOX5-like isoforms are also found in protists and plants, whereas insects, nematodes, and rodents do not express NOX5 (Bedard et al., 2007; Kawahara et al., 2007). In humans, NOX5 is expressed in lymphoid organs, testis, and spleen (Touyz et al., 2019).

DUOX1 and DUOX2 enzymes emerged from NOX5 by the addition of a peroxidase homology domain (Kawahara et al., 2007; Touyz et al., 2019). DUOX enzymes were first described to be involved in thyroid hormone biosynthesis as a source of hydrogen peroxide (Dupuy et al., 1999). This is in contrast to the other NOX family members that produce only superoxide. In addition to mammals, peroxidase activity of DUOX has been shown in the nematode *Caenorhabditis elegans* (Meitzler and Ortiz de Montellano, 2009; Morand et al., 2009). In humans, DUOX1 is expressed in the lung, salivary glands, pancreas, placenta, and testis (Edens et al., 2001), whereas DUOX2 is expressed in the trachea, stomach, colon, and rectum (Edens et al., 2001; Geiszt et al., 2003). In polarized cells, DUOX localizes to the apical plasma membrane (El Hassani et al., 2005; Forteza et al., 2005) and is involved in antimicrobial defense via hydrogen peroxide production in secretory glands and on mucosal surfaces (Geiszt et al., 2003).

### NOX in Phagocytes Across Different Species

NADPH oxidases family members fulfill distinct roles in various species. In the following, we will discuss the expression patterns of NOX orthologs across common model organisms to resolve the diverse function of these enzymes in phagocytes.

#### Nematodes

The nematode *C. elegans* is a powerful model organism to study the conserved host innate immune mechanisms, given that its genome was the first one to be entirely sequenced, its easy culturability under laboratory conditions, and the existence of conserved host–microbe interactions (Kumar et al., 2020). The NADPH oxidases in *C. elegans*, termed Ce-DUOX, consists of a gp91^phox^ homology region, and a peroxidase homology domain (Edens et al., 2001). The peroxidase domain forms two bonds with heme that have a catalytic function (Meitzler and Ortiz de Montellano, 2009). Ce-DUOX1 plays imperative roles in the protection against pathogens, e.g., *Enterococcus faecalis* (Chávez et al., 2007,2009) and *Candida albicans* (van der Hoeven et al., 2015). Less Ce-DUOX expression leads to decreased ROS production and increases susceptibility to *E. faecalis* (Chávez et al., 2009). ROS production activates SKN-1, an ortholog of the mammalian NRF transcription factor family, via p38 MAPK signaling (Van Der Hoeven et al., 2011).

#### Zebrafish

The study of zebrafish has provided new insights due to the availability of transgenic models of innate immunity disorders, combined with superior opportunities of *in vivo* imaging, given the transparency of the larvae (Harvie and Huttenlocher, 2015; Masud et al., 2019). Zebrafish express NOX1, NOX2, NOX4, NOX5, and a single isoform of DUOX (Kawahara et al., 2007). They possess all innate immune cell types and exhibit a similar functional diversity in phagocytes as mammals (Linnerz and Hall, 2020). NOX2 is expressed and functioning in both neutrophils and macrophages and transgenic lines are available to fluorescently label and genetically manipulate the specific subsets. As discussed below, p22^phox^-deficient larvae show increased susceptibility to fungal infection with excessive inflammation (Schoen et al., 2020).

#### Insects

Insects possess phagocytic cells, which engulf and kill pathogens under superoxide production (Browne et al., 2013). Plasmatocytes, the most common hemocytes, are macrophage-like cells similar to mammalian tissue macrophages (Buchon et al., 2014). In *Lepidoptera*, the cellular defense is mediated by plasmatocytes and granular cells, while in *Drosophila*, plasmatocytes and lamellocytes are key players (Browne et al., 2013). However, single-cell sequencing recently indicated that multiple populations and states of hemocytes exist (Tattikota et al., 2020), suggesting further functional diversity.

*Drosophila* has proven to be highly useful for studying the evolutionarily conserved innate immune system. This particularly concerns the gastrointestinal tract given the similarity to mammalian intestinal physiology and the less complex microbiota profile (Broderick and Lemaitre, 2012; Wang et al., 2014; Liu et al., 2017; Trinder et al., 2017). Gut infection in *Drosophila* induces rapid ROS production (Ha et al., 2005b). The two NADPH oxidase enzymes in *Drosophila*, which control intestinal microbes, are DUOX and NOX (Ha et al., 2005a). Microbiota-derived lactate leads to the activation of intestinal NOX (Iatsenko et al., 2018), while DUOX is activated through pathogen-derived uracil (Lee et al., 2013). It was shown that the two isoforms are present in different gut regions of *Drosophila* (Dutta et al., 2015; Iatsenko et al., 2018). Presumably, the two oxidase enzymes have distinct functions due to the different roles of lactate and uracil in host metabolism. In the intestine, DUOX-derived ROS are mainly involved in host defense, and regeneration, while NOX-derived ROS mediate epithelial renewal (Iatsenko et al., 2018).

Macrophage-like plasmatocytes are involved in the phagocytosis and encapsulation of pathogens (Fauvarque and Williams, 2011). Upon infection, a biphasic ROS response occurs (Myers et al., 2018). Initially, upon stimulation, all hemocytes, including non-phagocytic prohemocytes and crystal cells, mount a transient ROS response, which, in turn, influences plasmatocyte activation. Subsequently, after bacterial uptake, a strong ROS signal can be detected in phagocytes. The ROS responses in *Drosophila* are thus distinct in different cell types, with respect to timing, activation mechanisms, and functions. Potentially, the rapid ROS pulse is produced by mitochondria, and the later ROS response by the NADPH oxidase (Myers et al., 2018). However, further investigations are required to fully comprehend the mechanisms of these two ROS responses and their cell-type-specific effects. While regulatory NOX subunits were not found in *Drosophila* (Kawahara and Lambeth, 2007; Sumimoto, 2008), hemocytes of the Lepidopteran species *Galleria mellonella* contain proteins homologous to p67^phox^ and p47^phox^, which translocate upon PMA stimulation (Bergin et al., 2005; Renwick et al., 2007).

#### Mammals

Most mammalian species express seven NOX isoforms: NOX1–5 and DUOX1–2. Rodents are an exception, as they do not possess NOX5 (Sumimoto, 2008). NOX2 is expressed in mononuclear phagocytes as well as all three types of granulocytes, i.e., neutrophils, eosinophils, and basophils (Buvelot et al., 2016). Phagocytes can release ROS both into the phagosome and the extracellular space due to expression of NOX2 on both the phagosomal and the plasma membrane, while eosinophils express it only on the plasma membrane (Holmdahl et al., 2016). B lymphocytes also express NOX2, albeit at lower levels (Holmdahl et al., 2016).

Similar gene loci and protein sizes for the different subunits of NOX2 have been identified in humans and mice. The *Cybb* gene that encodes gp91^phox^ is localized on chromosome Xp21.1. The molecular size of the gp91^phox^ protein in humans and rodents is similar, approximately 65.3 kDa (Lambeth et al., 2000). In humans, the chromosomal position of the *Ncf1* gene, which encodes p47^phox^, is 7q11, whereas in mice, it resides in the distal region of chromosome 5, in a region of high homology to human 7q11. While the mouse gene shows a reduced size, the number of exons and introns are conserved and exons exhibit a high degree of sequence homology (DeSilva et al., 2000).

### Activation of Phagocyte NOX

The activation of the mammalian phagocyte NOX is tightly regulated and predominantly depends on the engagement of surface receptors by dedicated ligands. Subsequent to their activation, enzymatic subunits assemble at the membrane (Figure 2). The gp91^phox^ subunit provides a conserved electron transportation region and NADPH and FAD binding sites. It forms, together with p22^phox^, the catalytic core, a non-covalent heterodimer that resides at phagosomal, granule, and the plasma membrane. The regulatory subunits p67^phox^, p47^phox^, and p40^phox^ reside in the cytoplasm as complex. Upon stimulation, p47^phox^ undergoes phosphorylation, and the complex translocates to the membrane along with the small GTPase Rac2 in order to activate flavocytochrome b_558_ (Lambeth, 2004; Nauseef, 2004; Sumimoto et al., 2005). The underlying molecular events have recently been reviewed in detail (Brandes et al., 2014; Nguyen et al., 2017; Belambri et al., 2018).

**FIGURE 2:** Activation and assembly of mammalian NOX2. NOX2 consists of the cytosolic components p67^phox^, p47^phox^, p40^phox^, Rac2, and the integral membrane subunits gp91^phox^ and p22^phox^. Upon cell stimulation, the cytosolic subunits translocate to the membranes to form an active complex with gp91^phox^ and p22^phox^. Meanwhile, Rac exchanges GDP to GTP, and dissociates from Rho-GDI. In the resting state, the p47^phox^-SH3 tandem domain interacts with AIR keeping p47^phox^ in an inactive conformation (Belambri et al., 2018). Cell stimulation induces phosphorylation of AIR, releasing the interactive domains, i.e., SH3, PX, and PRR, which mediate oxidase assembly. The PRR of p47^phox^ binds to the SH3 region of p67^phox^, while p67^phox^ links with p40^phox^ through their PB1 domains. The p47^phox^-SH3 regions then bind to the p22^phox^-PRR domains promoting p67^phox^ interaction with gp91^phox^ and moving p40^phox^-PX domains in close proximity to the membrane. Activated NOX2 uses cytosolic NADPH to induce oxygen reduction and superoxide anion (O_2_⋅-) generation. Abbreviations: SH3, Src homology 3 (SH3);, PX, phox homology (PX);, AIR, auto-inhibitory region (AIR);, PRR, proline-rich region (PRR);, TPR, tetratricopeptide-rich regions; PB1, phox and Bem1 domain; and AD, activation domain.

Some cell surface receptors, including Toll-like receptors (TLRs), G-protein-coupled receptors (GPCRs), and TNF receptors (TNFRs), can prime the phagocytes for NOX2 activation (Nguyen et al., 2017). Priming may include conformational changes or partial phosphorylation of the regulatory subunits, which renders the cells more susceptible to a secondary stimulus but does not lead to superoxide production. Stimulation of other receptors, including Fc and integrin receptors, and the GPCR recognizing *N*-Formylmethionine-leucyl-phenylalanine (fMLP) result in direct activation of NOX2 (Nguyen et al., 2017). Their interaction with enzymes such as phospholipase C leads to the activation of protein kinase C (PKC) family members, which phosphorylate the cytosolic subunits of NOX2. PMA, on the other hand, penetrates the plasma membrane and directly induces PKCα and β activation and phosphorylation of p47^phox^ (Fontayne et al., 2002). The p47^phox^ subunit harbors a tandem Src homology 3 (SH3), an auto-inhibitory region (AIR), and a proline-rich region (PRR) at the C-terminus (Figure 2). A phosphoinositide-interacting PX domain in the N-terminus mediates binding to phosphoinositides [PI(3,4)P2] of the plasma membrane (Hiroaki et al., 2001). In the cytoplasm of resting phagocytes, the SH3 domains are blocked due to the intramolecular interaction with AIR. Upon stimulation, phosphorylation leads to the release of the PRR/AIR domain and the open structure can bind to the other subunits (Yuzawa et al., 2004; Minakami and Sumimoto, 2006). The SH3 domain then binds to p22^phox^ of flavocytochrome b_558_ and the PX domain to the plasma membrane, bringing p67^phox^ in close proximity to Nox2. The p67^phox^ subunit contains an activation domain in the center, which subsequently activates NOX2.

The third component of the cytosolic complex, p40^phox^, contains a PX domain that mediates binding to phosphatidylinositol-3-phosphate [PI(3)P] in phagosomal membranes (Suh et al., 2006). This binding domain was shown to be essential for oxidase activation in response to fungal particles in human, but not mouse neutrophils (Bagaitkar et al., 2012). Consequently, mouse neutrophils do not depend on p40^phox^ for NOX activation. In addition, p40^phox^-deficient patients show a selective loss of NOX activity in response to ingested particles in neutrophils, but not mononuclear phagocytes (van de Geer et al., 2018). Accordingly, mouse macrophages and monocytes may also be capable of signaling independently of p40^phox^. Finally, Rac, a member of the Rho family of small GTPases, critically regulates the oxidase activity (Miyano and Sumimoto, 2012). The isoform Rac1 is ubiquitously expressed, while Rac2 is only expressed in hematopoietic cells where it is mainly responsible for NOX2 activation (Panday et al., 2015). The inactive form is bound to GDP and Rho-GDI, the GDP dissociation inhibitor. In response to stimulation, GDP is converted to GTP, mediating dissociation of Rho-GDI and Rac translocation.

### ROS as Signaling Molecules

Reactive oxygen species are involved in a range of cellular and tissue responses. Additionally, ROS derived from different NOX influence distinct downstream signaling pathways, which may be the reason for co-expression of more than one isoform of NOX in specific cell types (Dworakowski et al., 2006). Upon NOX assembly, electrons are shuttled from cytosolic NADPH to FAD to membrane-embedded heme groups, which then reduce molecular oxygen to superoxide (O_2_^–^). The superoxide anion is a highly reactive “non-diffusible” state that is spontaneously or enzymatically converted to hydrogen peroxide (H_2_O_2_). In granulocytes, H_2_O_2_ is rapidly transformed to bactericidal hypochlorous acid (HOCl) via the action of the granule-contained myeloperoxidase (Chen et al., 2011; Nguyen et al., 2017). H_2_O_2_, on the other hand, is a stable “diffusible” oxidant, which may induce cytoplasmic signaling molecules (Gough and Cotter, 2011).

Reactive oxygen species play a role in various signaling pathways as second messenger. They can influence MAPK cascades and calcium signaling via oxidation of signaling intermediates (Zhang et al., 2016), and may affect cellular proliferation as well as cell death (Lambeth, 2004; Morgan and Liu, 2010; Schenk and Fulda, 2015). ROS can regulate actin and microtubule dynamics due to the oxidation of certain amino acid residues in microtubules and actin microfilaments (Wilson and González-Billault, 2015). H_2_O_2_ can promote cell migration through the regulation of actin dynamics and cytoskeleton organization (Kim et al., 2009). The release of DUOX-derived H_2_O_2_ by the zebrafish epithelium attracts leukocytes to the wound (Niethammer et al., 2009). In human, ROS are critical for wound healing via induction of thrombus formation; recruitment of peripheral blood cells, endothelial cells, keratinocytes, and fibroblasts; and promotion of cell division (Lambeth, 2004; Dunnill et al., 2017). Generally, the effects of ROS strongly depend on the amount, source, reactivity, and half-life of the produced ROS and the cellular compartment of its production. In the following, we will thus focus on effects of ROS generated by phagocytes and emphasize on the source of ROS wherever possible, e.g., through the use of genetically deficient animals or patients with CGD, where monogenetic aberrations abrogate ROS formation (see below).

### Expression of NOX Homologs in Phagocytes

Apart from NOX2 expression in phagocytes, it has been reported that NOX1 (Maitra et al., 2009), NOX4 (Lee et al., 2010), and NOX5 (Marzaioli et al., 2017) are also expressed in phagocytes. In murine macrophages, stimulation with LPS leads to activation of NOX1. IRAK-1, downstream intracellular signaling components of TLR4, induces the transcription of NOX1 via NF-κB and other related transcription factors (Maitra et al., 2009). In addition, NOX1 was shown to play a role together with NOX2 in M2 polarization and macrophage differentiation by induction of the JNK and ERK signaling pathways (Xu et al., 2016). NOX4, on the other hand, localizes to the endoplasmic reticulum and mediates intracellular ROS generation in human monocytes and mature macrophages (Lee et al., 2010). Furthermore, NOX4 contributes to the polarization of macrophages. It appears to have an anti-inflammatory role in macrophages, as NOX4 deficiency favors the polarization of proinflammatory human macrophages and promotes NF-κB activity (Helfinger et al., 2019). Furthermore, expression of NOX1 (Chéret et al., 2008) and NOX4 (Li et al., 2009) was shown in microglia.

Finally, NOX5 expression was detected in the THP-1 cell line and primary CD14^+^ human monocytes (Manea et al., 2015). Immunohistochemical staining data confirmed the presence of the NOX5 in CD68^+^ macrophages. A recent publication demonstrated that NOX5 expression is strongly increased during the differentiation of monocytes into dendritic cells (DCs), but not macrophages (Marzaioli et al., 2017). Additionally, NOX5 expression was detected in circulating myeloid DC. Mechanistically, the NOX5–p22^phox^ complex mediates DC differentiation from monocytes through regulation of the JAK/STAT/MAPK and NF-κB pathways (Marzaioli et al., 2017). Collectively, these studies demonstrate that phagocytes may express other NOX isoforms except for NOX2 at certain developmental stages and after polarization. The relative contribution of these alternative ROS sources remains unclear at this stage. However, they should be considered in situations when regulatory subunits are lost, such as p22^phox^ with functions in several isoforms, or general ROS inhibitors are used for investigations in phagocytes.

### NOX-Independent ROS Formation by Phagocytes

Next to NOX, cell organelles may contribute to ROS formation in phagocytes. Mitochondria are the main ROS source besides NOX in mammals, while the endoplasmic reticulum and peroxisomes are less important. In mitochondria, superoxide anions are produced during oxidative phosphorylation by reduction of molecular oxygen, which are further converted to H_2_O_2_ by superoxide dismutases (Hamanaka and Chandel, 2010). Mitochondria can produce ROS (mtROS) in a TLR-dependent fashion and are recruited to macrophage phagosomes (West et al., 2011). MtROS-derived H_2_O_2_ may then be directly delivered to bacteria-containing phagosomes via mitochondria-derived vesicles (Abuaita et al., 2018). These mechanisms can directly contribute to bactericidal activity in macrophages. In zebrafish, it was shown that macrophages use fatty acid β-oxidation in infection to produce mtROS, which is regulated via Irg1 (immunoresponsive gene 1) (Hall et al., 2013). For *Drosophila*, the impact of mtROS on the innate immune response is less clear. Biphasic ROS production after bacterial infection may suggest that hemocytes produce mitochondrial and enzyme-derived ROS upon infection as well (Myers et al., 2018). While macrophages can produce high amounts of mtROS, especially after stimulation, neutrophils contain only low numbers of active mitochondria (Dupre-Crochet et al., 2013).

A cross-talk between NOXs-derived ROS and mitochondria, which was termed “ROS-induced ROS release,” may amplify ROS generation at different subcellular compartments (Fukai and Ushio-Fukai, 2020). NOX4-derived H_2_O_2_ may augment mtROS, which could be limited by NOX2 siRNA (Kim et al., 2017). It was thus suggested that NOX2 can sense H_2_O_2_ and regulate mtROS generation (Kim et al., 2017). In addition, NOX-derived H_2_O_2_ of phagocytes can stimulate NOX in non-phagocytic cell types in a positive feedback loop to generate more oxidant species, which may be involved in vascular cell injury (Li et al., 2001). In addition to cell organelles, ROS may be produced in small amounts as a by-product in other enzymatic reactions, e.g., in the cytoplasm. The different sources of ROS were reviewed in more detail elsewhere (Dupre-Crochet et al., 2013).

## Functional Roles of Nox-Derived Oxidants in Phagocytes

### Myeloid Lineage-Specific Aspects

Phagocyte lineages differ in NOX2 expression and activity. After activation, neutrophils produce more ROS compared to monocytes and macrophages (Nauseef, 2019). DCs express little NOX2 and accordingly less ROS after activation (Mantegazza et al., 2008). In neutrophils, generation of H_2_O_2_ in the phagosomes activates myeloperoxidase in primary granules, which catalyzes the production of the highly antimicrobial and oxidative hypochlorous acid (Nguyen et al., 2017; Nauseef, 2019). Moreover, neutrophils are recruited to wounds via tissue-derived H_2_O_2_ and the myeloperoxidase was shown to clear H_2_O_2_ at the wound site in zebrafish (Yoo et al., 2011; Pase et al., 2012; Linnerz and Hall, 2020). Additionally, NOX2 activates granular proteases and triggers the generation of neutrophil extracellular traps (NETs) (Singel and Segal, 2016; Nguyen et al., 2017). These filamentous protein and chromatin structures are released extracellularly and aid in killing extracellular bacteria. Neutrophils of CGD patients are incapable of NETosis, which was restored by gene therapy in a CGD patient (Bianchi et al., 2009). NET formation was also absent in lungs of p47^phox^-deficient mice after *Aspergillus* infection (Röhm et al., 2014). As excessive neutrophil activity after infection may cause tissue damage, cell death of activated neutrophils is physiologically important and tightly regulated. In the context of infection, this process, termed pathogen-induced cell death, depends on NOX activity (Lawrence et al., 2020). Impaired NETosis and reduced efferocytosis may thus contribute to the overall hyperinflammatory phenotype in CGD patients. As neutrophils contain only few mitochondria, the impact of mtROS is considered to be low (Dupre-Crochet et al., 2013).

Mononuclear phagocytes, on the other hand, do not express myeloperoxidase and thus contain more H_2_O_2_ in their phagosomes (Nauseef, 2019). In addition, mitochondrial H_2_O_2_ is delivered to phagosomes (Abuaita et al., 2018). As ROS production is a hallmark of classically activated M1 macrophages, ROS are essential for induction and function of the M1 phenotype (Mills and O’Neill, 2016; Rendra et al., 2019). However, it was found that superoxide is also produced during alternative macrophage activation and that the inhibition of ROS blocks the polarization to M2 macrophages (Zhang et al., 2013). Yet, since the inhibitors, which were employed in this study, also interrupted mitochondrial ROS, the source of ROS remained unclear. Another study found that M2 polarization is impaired in macrophages with a combined deficiency in NOX1 and 2, which was connected to wound healing deficits (Xu et al., 2016). Overall, it is not yet clear how polarization of macrophages is influenced by ROS, as it likely depends on several parameters including phagocyte differentiation stage and source of ROS. Similarly, it is not understood how ROS affect the differentiation of tissue macrophages. At least in the murine brain, NOX2 is activated during the development of microglia, the resident macrophages, and promotes their infiltration into the subventricular zone of the cerebral cortex (Lelli et al., 2013).

P47-deficient mice, which were complemented with a functional allele of p47 only in CD68+ cells (i.e., monocytes and macrophages), were shown to be more resistant to staphylococcal and *Aspergillus* infection, indicating that NOX2 in mononuclear phagocytes is crucial in the systemic defense against bacteria and fungi (Pizzolla et al., 2012; Grimm et al., 2013). Moreover, patients with a macrophage-specific mutation in *Cybb* (gp91^phox^) are particularly prone to mycobacterial disease (Bustamante et al., 2011). In these patients, a germline mutation in the *Cybb* allele impairs NOX assembly and respiratory burst in macrophages, but not in monocytes and neutrophils. Accordingly, the assembly of NOX depends on cell-specific thresholds.

NOX2 is also expressed in DCs, albeit at lower levels. In these cells, the enzyme is recruited to early phagosomes where it utilizes protons for ROS production, thereby limiting acidification of the phagosomes. In the absence of NOX2, phagosomes of mouse DCs show decreased proteolysis and consequently degradation of antigen, resulting in impaired antigen cross-presentation skills (Savina et al., 2006; Rybicka et al., 2012). Cross-presentation of tumor antigens is also impaired in DCs from human CGD patients (Mantegazza et al., 2008). In contrast, the acidification of phagosomes of macrophages, which exhibit much higher NOX2 activity, is positively affected by ROS production (Bagaitkar et al., 2018). In efferocytosis, phagosomes of peritoneal macrophages of CGD mice showed delayed maturation and acidification, resulting in decelerated disposal of apoptotic cells (Bagaitkar et al., 2018). In addition, cross-presentation of antigens was increased in these cells. The opposed function of NOX2 in macrophages and DCs might relate to the higher expression of the V-ATPase and lysosomal proteases in macrophages.

### Cell-Intrinsic Effects

The functions of NOX2 and of NOX2-derived oxidants can generally be subclassified in effects on the individual cell level and the population/tissue level. Effects due to autocrine signaling occur in the individual phagocyte after NOX2 activation.

Neutrophils of CGD patients show globally increased expression of proinflammatory mediators in steady state (Kobayashi et al., 2004). In response to toll-like receptor ligands, human and mouse leukocytes exhibit increased production of proinflammatory cytokines such as IL-6 and TNF along with elevated NF-κB activation (Bylund et al., 2007; Brown et al., 2008). Notably, increased expression of inflammatory cytokines has also been described in p22^phox^-deficient larvae of zebrafish in steady state as well as in response to fungal infection (Schoen et al., 2020). In the past, the activation of NOX2 was linked to the activation of the inflammasome, multimeric cytosolic pathogen sensors. According to some earlier studies, NOX2-derived ROS were described as essential second stimuli for the activation of the NLRP3 inflammasome (Dostert et al., 2008). However, it was later shown that the NLRP3 inflammasome does not depend on NOX1–4-derived ROS for its activation (van Bruggen et al., 2010), but instead on mitochondrial ROS (Zhou et al., 2011; Netea et al., 2015). On the contrary, monocytes from CGD patients exhibited increased caspase activation and IL-1β secretion in comparison to controls (Meissner et al., 2010; van de Veerdonk et al., 2010). de Luca et al. (2014) showed that macrophages from CGD mice and monocytes from CGD patients were deficient in autophagy, leading to increased IL-1β release after stimulation. Blockage of the IL-1β receptor limited inflammasome activation and restored autophagy, resulting in decreased neutrophil recruitment and amelioration of colitis in some CGD patients. Thus, NOX2 appears to be important for the negative regulation of IL-1β-dependent signaling. Moreover, NOX2-derived ROS are involved in the induction of a non-canonical autophagy pathway, called LC3-associated phagocytosis (LAP) (Huang et al., 2009; de Luca et al., 2014; Martinez et al., 2015). In LAP, components of the autophagy pathway, i.e., LC3, are targeted to phagosomal membranes, leading to efficient fusion with lysosomes and destruction of contained pathogens. Notably, this pathway is particularly important for the clearance of *Aspergillus fumigatu*s, which often causes invasive infections in CGD patients.

Additionally, the hyperinflammatory phenotype in CGD has been linked to defective tryptophane metabolism, as the kynurenine pathway, the major pathway for tryptophane degradation, was supposedly dependent on superoxide (Romani et al., 2008). However, several later studies found tryptophan catabolism to be normal in NOX2-deficient patients and mice (De Ravin et al., 2010; Jürgens et al., 2010; Maghzal et al., 2014). The increased cytokine expression in response to stimuli in CGD was instead traced back to impaired activation of the nuclear factor erythroid 2-related factor 2 (Nrf2), a key redox-sensitive transcription factor (Segal et al., 2010). Nrf2 regulates oxidative stress pathways and acts anti-inflammatory by suppressing the transcription of proinflammatory cytokines (Kobayashi et al., 2016). Consequently, mononuclear cells from peripheral blood from CGD patients show reduced Nrf2 activity and increased NF-κB activation (Han et al., 2013; Singel and Segal, 2016). Furthermore, it was suggested that NOX2 deficiency promotes nuclear accumulation of thioredoxin-1, an antioxidant protein with a disulfide reductase activity (Trevelin et al., 2016). Thioredoxin-1 in turn contributes to the DNA binding of NF-κB subunits by posttranslational modification (Matthews et al., 1992; Trevelin et al., 2016; Muri et al., 2020). Thus, the activity of NOX2 may influence the NF-κB pathway via interaction with multiple nuclear proteins, ensuring the regulation of proinflammatory cytokines. These processes are largely conserved from zebrafish to mammals.

In general, ROS derived from mitochondria contribute to cellular signaling as well. MtROS contribute to proinflammatory cytokine secretion by disulfide linkage of the essential modulator of NF-κB NEMO (Herb et al., 2019) and stimulate the activation of the NLRP3 inflammasome (Zhou et al., 2011). Thus, the effect of ROS on cytokine secretion depends additionally on the cellular source and localization of ROS. In line with that, a recent study suggested that mtROS are elevated in CGD phagocytes, which paradoxically leads to oxidative stress and increased MAPK activation and may thus further contribute to production of proinflammatory cytokines (Sundqvist et al., 2017).

### Cell-Extrinsic Effects

The assembly of NOX2 at the plasma membrane allows for the production of extracellular ROS intermediates (Nauseef, 2019). Production of extracellular H_2_O_2_ may thus affect cells of the surrounding tissue. In general, NOX2 is recognized to play an important role in the calibration of the immune response, i.e., to limit inflammatory responses after injury or infection (Singel and Segal, 2016). This effect may be achieved by dampening of the IL-1β response in macrophages, thereby leading to the recruitment of less neutrophils (de Luca et al., 2014). The effect of ROS also depends on the production site. Warnatsch et al. (2017) showed that neutrophils produced intracellular ROS in mice infected with small microbes, while ROS were secreted into the extracellular space in infection with large microbes such as filamentous fungi. Intracellular ROS suppressed IL-1β expression in these neutrophils, thus limiting recruitment of additional neutrophils, while extracellular ROS amplified IL-1β secretion and neutrophil clustering. Hence, the assembly of NOX2 on the phagosomal or the plasma membrane impacts on the outcome of the entire tissue reaction.

Secondly, the production of large quantities of superoxide during the respiratory burst may lead to the depletion of oxygen in the surrounding tissue, e.g., in the context of acute colitis. Transmigrating neutrophils rapidly deplete microenvironmental oxygen in the lamina propria, leading to stabilization of the hypoxia-inducible factor HIF and HIF-dependent responses in intestinal epithelial cells (Campbell et al., 2014). Furthermore, gp91^phox^-deficient mice showed increased infiltration of granulocytes, but diminished hypoxia and worsened colitis. Thus, the NOX2-dependent modulation of extracellular oxygen may be protective in colitis, due to activation of hypoxic responses in neighboring cells, highlighting the complexity of ROS signaling on the tissular level.

Recently, a paracrine effect of NOX2 was shown to facilitate interaction between neutrophils and macrophages after liver injury (Yang et al., 2019). Genetic deficiency in gp91^phox^ delayed liver recovery, due to a failure of pro-inflammatory Ly6C^hi^CX_3_CR1^low^ macrophages to convert into pro-resolving Ly6C^low^CX_3_CR1^high^ macrophages. Adoptive transfer of WT, but not gp91^phox^-deficient neutrophils, rescued the conversion in neutropenic mice. Thus, NOX2-derived ROS from neutrophils appear to shape the phenotype of tissue macrophages and thereby orchestrate tissue repair. A ROS-dependent bidirectional communication was also observed between hemocytes, the macrophages of *Drosophila*, and epithelial cells (Fogarty et al., 2016). Extracellular DUOX-derived ROS formed by epithelial cells led to macrophage activation, which in turn triggered apoptosis-induced proliferation in epithelial cells via TNF. Accordingly, the diffusion of ROS and in particular H_2_O_2_ within the tissue or even across membranes (Nauseef, 2019; Yang et al., 2019) may influence signaling and cellular processes of other cell types within the same tissue or even across membranes in distant tissues. In *Drosophila*, increased levels of ROS sensitize hematopoietic progenitors to differentiate into mature innate blood cells (Owusu-Ansah and Banerjee, 2009), and after parasite infection, induction of ROS in hematopoietic cells leads to secretion of epidermal growth-factor like cytokine resulting in differentiation of specialized innate immune cells (Sinenko et al., 2012). Consistent with this model, hematopoietic stem cells were found to be diminished in bone marrow and peripheral blood of CGD patients (Weisser et al., 2016).

NOX2 might also affect adaptive immunity. A type 1 interferon signature was found in CGD mice and patients, accompanied by the presence of autoantibodies, pointing toward autoimmune features of NOX2 deficiency (Kelkka et al., 2014). Notably, CGD patients exhibit an increased frequency of autoimmune diseases (Schäppi M. G. et al., 2008). Female carriers of X-linked CGD with varying degrees of inactivation in the mutated X chromosome also show autoimmune manifestations, which, in some cases, included lupus-like symptoms (Cale et al., 2007; Marciano et al., 2018). In mice, gp91^phox^ deficiency led to a heightened susceptibility for autoimmune arthritis (George-Chandy et al., 2008). Generally, the increased expression of proinflammatory cytokines may enhance T cell activation by antigen-presenting cells (George-Chandy et al., 2008). In addition, NOX2-deficient rat and human macrophages are less capable to induce regulatory T cells (Kraaij et al., 2010). For more details on the impact of ROS on lymphocyte signaling, we refer the reader to recent reviews (Cachat et al., 2015; Holmdahl et al., 2016). Altogether, NOX2-derived ROS may shape the regulation of the adaptive immune response and play a role in the resolution of the inflammatory response. The mechanisms discussed in the previous paragraph, such as enhanced secretion of proinflammatory mediators and decelerated disposal of apoptotic cells may contribute to this effect.

## Phagocyte-Derived ROS in Health and Disease

In general, ROS are recognized to play a role in physiological as well as pathological states and the literature covering this subject has increased extensively. While NOX-derived ROS are important for basic physiological functions such as the regulation of blood pressure and gut motility, excess ROS may promote cellular stress and contribute to the development of autoimmunity or cancer (Sorescu et al., 2002; Block and Gorin, 2012; Gray Stephen et al., 2013; Nayernia et al., 2013; Panday et al., 2015; Konaté et al., 2020). As an example, it was found that in acute myeloid leukemia, NOX-derived ROS promote proliferation of leukemic cells (Hole et al., 2013). For the present review, we will finally focus on two aspects directly related to the expression of NOX in phagocytes, i.e., the interplay with the microbiota and the clinical perspective of CGD.

### The Specific Role of NOX in the Cross-Talk With the Microbiota

In steady state, NOX-derived ROS are involved in the interspecies cross-talk with the individual microbiota. This has been exemplified in *Drosophila*, which exhibits a low degree of bacterial diversity in the microbiota (Wong et al., 2011). Both in fruit flies and mice, commensal bacteria induce NOX1-dependent ROS and thereby stimulate the proliferation of intestinal stem cells (Jones et al., 2013). In contrast, an overgrowth of commensals with increased formation of lactic acid induces excessive intestinal NOX activity and ROS production, and, as a result, intestinal damage in *Drosophila* (Iatsenko et al., 2018). The underlying mechanism is the oxidation of lactate by the host lactate dehydrogenase, which produces NADH for NOX, uncovering a metabolic cross-talk between microbiota and host with contribution by ROS. Analogous mechanisms in mammals involve symbionts inducing ROS generation by intestinal epithelial cells, thereby impacting on host physiology (Jones and Neish, 2017). In contrast, few studies have investigated the direct impact of phagocytic NOX on the host–microbiome interaction. In p47^phox^-deficient mice, susceptibility for DSS colitis was reversed by standardizing the microflora from birth on (Falcone et al., 2016), indicating that impaired NOX2 activity might have a lasting impact on the microbiome composition. In case the microbiome is disturbed by antibiotics, NOX2 is required for host survival in a *Citrobacter rodentium* infection model (Pircalabioru et al., 2016; Knaus et al., 2017). Thus, the commensal microbiota may act in concert with NOX2 to protect the intestine from the invasion of virulent microorganisms.

In patients suffering from CGD, the spectrum of microbes causing infections is surprisingly narrow, indicating which pathogens are targeted in particular by NOX2. Patients frequently present with severe fungal infections, especially by *Aspergillus* spp., which also account for most infection-related deaths in CGD (Henriet et al., 2012; Marciano et al., 2015). Next to the prevalent *A. fumigatus*, *Aspergillus nidans* imposes a specific risk pathogen in CGD patients, which is uncommon in other immunodeficiencies (Henriet et al., 2012). Interestingly, zebrafish larvae with p22^phox^-deficiency are also more susceptible to *Aspergillus nidulans* infection with enhanced inflammation, which was attributed to both excessive neutrophil recruitment as well as fungal growth (Schoen et al., 2020). Potentially, increased inflammation caused by this normally avirulent fungus results in its fast clearance but, in case of CGD deficiency, leads to detrimental inflammatory damage to the host instead.

With regard to bacteria, *Staphylococcus*, *Burkholderia*, and *Serratia* are leading causes of infection in CGD (Marciano et al., 2015). Similarly, NOX2-deficient rodents show increased susceptibility to *Staphylococcus aureus* and *Aspergillus* (Pollock et al., 1995; Pizzolla et al., 2012; Grimm et al., 2013). In a cohort of 268 patients, about one third suffered from severe infections with *S. aureus*, which was isolated from lymph nodes and liver abscesses (Marciano et al., 2015). Notably, neutrophils of CGD patients show a decreased capacity to kill *S. aureus* but not *Escherichia coli* (Rosen and Michel, 1997). It is not entirely clear why NOX2 is particularly important in the defense against *S. aureus*, as the bacterium possesses multiple resistance mechanisms such as catalase and superoxide dismutase (Buvelot et al., 2016). Next to the direct killing capacity, ROS may directly modify staphylococcal gene regulation (Rothfork et al., 2004; Buvelot et al., 2016). On the other hand, the regulation of the immune response by NOX2, in particular the inflammatory response as discussed above, may be essential to eliminate *S. aureus*. Also in *Aspergillus*, antioxidant pathways may overcome direct damage by ROS (Lambou et al., 2010; Wiemann et al., 2017; Schoen et al., 2020). This demonstrates a large degree of adaptation by the pathogens, which are particularly affected by this host defense mechanism. Thus, next to direct damage of bacterial DNA or proteins, the control and regulation of the inflammatory response may be equally important in the containment of these pathogens.

Finally, CGD patients show an increased susceptibility for mycobacteria, i.e., *Mycobacterium tuberculosis* in endemic countries and *Mycobacterium bovis* (BCG) after vaccination (Deffert et al., 2014; Conti et al., 2016). As mentioned above, patients with a macrophage-specific mutation in *Cybb* are particularly prone to mycobacterial disease (Bustamante et al., 2011). P47^phox^-deficient mice also show increased growth of *Mycobacterium tuberculosis* in the lungs at early stages of pulmonary infection (Cooper et al., 2000). Moreover, NOX-dependent mechanisms are essential for neutrophil-mediated killing of *Mycobacterium marinum* in zebrafish larvae after granuloma formation (Yang et al., 2012). Thus, oxidative killing of mycobacteria is a conserved mechanism by which phagocytes protect their respective hosts.

In addition to monogenetic and deleterious aberrations, single-nucleotide polymorphisms and hypomorphic mutations in *Nox* subunit genes have been associated with increased risks for IBD (Dhillon et al., 2014; Aviello and Knaus, 2018). IBD, on the other hand, is often associated with dysbiosis. Yet, it is unclear if this is causal for or a result of increased inflammation. As almost every second CGD patient suffers from intestinal inflammation (Marks et al., 2009; Falcone et al., 2016), further research is needed on the role of NOX2 in intestinal integrity, in particular in terms of local immune homeostasis and the microbiota.

### CGD: Clinics and Animal Models

Chronic granulomatous disease is an immunodeficiency disease caused by defects in any of the five structural components of the NOX enzyme, i.e., X-linked recessive mutations in *Cybb* (gp91^phox^), or autosomal recessive mutations in *Cyba* (p22^phox^), *Ncf1* (p47^phox^), *Ncf2* (p67^phox^), or *Ncf4* (p40^phox^) (Kuhns et al., 2010; Arnold and Heimall, 2017; van de Geer et al., 2018). Gp91^phox^-deficient CGD is the most common and severe form of this disease in human (Kuhns et al., 2010). Gp91^phox^-deficient patients produce very low amounts of ROS, while neutrophils in patients with mutations in *Ncf1* form higher amounts, leading to an overall increased survival rate. Recently, a novel cause for CGD was discovered in patients with a deficiency in the *Cybc1* gene (Arnadottir et al., 2018; Thomas et al., 2019). Cybc1 encodes the ER-resident protein EROS (Essential for Reactive Oxygen Species), which is required for stable expression of the gp91^phox^ and p22^phox^ proteins and putatively acts as chaperone for the heterodimer in humans and mice (Thomas et al., 2017; Arnadottir et al., 2018).

The CGD incidence is between 1 in 200,000–250,000 newborns in Europe and the United States (Winkelstein et al., 2000; Arnold and Heimall, 2017). As described in the previous paragraph, invasive bacterial and fungal infections are pivotal contributors to morbidity and mortality in CGD patients. Bacterial infections typically affect the lungs, skin, liver, and lymph nodes (Arnold and Heimall, 2017). Dysregulated inflammation on the other hand most commonly affects the gastrointestinal tract, followed by lungs, urogenital tract, and eyes. In addition, liver abnormalities including nodular regenerative hyperplasia and non-cirrhotic portal hypertension have been observed in NOX2-deficient patients (Hussain et al., 2007). In gp91^phox^-deficient individuals, inflammatory complications occur twice as often as in patients with autosomal recessive NOX gene mutations (Arnold and Heimall, 2017). Moreover, X-linked CGD patients exhibit a strong and early disease phenotype, and an earlier age of death (van den Berg et al., 2009).

Granuloma formation is a typical CGD manifestation (Schäppi M. G. et al., 2008). Granulomas can occur in various organs such as colon, lung, and skin and may functionally impair the respective organs. While granulomas can form as a reaction to chronic infection, they may also form in the absence of overt infection, i.e., the absence of cultivable microbes. In CGD patients, their response to immunosuppressants rather than antibiotics clearly indicates immunodysregulation (Schäppi M. G. et al., 2008). In NOX2-deficient mice, persistent inflammatory lesions develop in response to sterile preparations of fungal cell walls in the lung and skin (Morgenstern et al., 1997; Schäppi M. et al., 2008). Furthermore, mice deficient in *Ncf1* or *Cyba* were reported to develop spontaneous granulomas in the lung, even if housed under SPF conditions (van der Weyden et al., 2018). Thus, granulomatous lesions in CGD patients may not just deflect impaired microbial killing, but rather the dysregulation of the inflammatory response and the failure to efficiently clear debris.

The CGD models in zebrafish comprise deficiencies in gp91^phox^ and p22^phox^. CGD zebrafish models are susceptible to *Pseudomonas aeruginosa* and to *A. nidulans* (Henriet et al., 2012; Yang et al., 2012). Additionally, excessive neutrophil recruitment is observed (Schoen et al., 2020). Both the fungal growth and the neutrophilic inflammation could be limited by expression of NOX in neutrophils alone, indicating that the aberrant signaling in neutrophils contributes to both higher microbial susceptibility and the hyperinflammatory phenotype in zebrafish (Schoen et al., 2020).

Around 50% of patients with CGD suffer from severe intestinal inflammation, which shares features with inflammatory bowel disease (IBD), according to a report of the National Institutes of Health (Falcone et al., 2016). The gastrointestinal manifestations show striking similarities with Crohn’s disease (Marks et al., 2009) and mostly affect the colon, which shows microgranulomas, pigmented macrophages, and tissue eosinophilia (Alimchandani et al., 2013).

To understand the mechanisms of colitis in NOX2 deficiency, animal models have been extensively used. In NOX2-deficient mice, however, colitis does not develop spontaneously and requires induction, most commonly achieved by chemicals. In the trinitrobenzenesulfonic acid (TNBS) model, colitis is stimulated via T lymphocyte responses due to haptenization of host or microbiota-derived proteins (Antoniou et al., 2016). Dextran sulfate sodium (DSS) treatment, on the other hand, exhibits toxicity against of intestinal epithelial cells, which stimulates disintegration of the mucosal membrane (Perše and Cerar, 2012; Wirtz et al., 2017). Thus, while the DSS model represents a wound model, the TNBS model is considered an acute-to-chronic inflammation model (Campbell and Colgan, 2019). For CGD, it was demonstrated that gp91^phox^-deficient mice are susceptible to the TNBS colitis model (Campbell et al., 2014). In contrast, DSS did not efficiently induce colitis in gp91-deficient mice; weight loss and colitis severity were less pronounced than in wild-type mice (Bao et al., 2011; Aviello et al., 2019). In addition, it was suggested that mice with gp91^phox^ deficiency also do not develop severe colitis after *C. rodentium* infection (Fattouh et al., 2013). Conversely, p47^phox^-deficient mice developed strong disease after DSS administration (Rodrigues-Sousa et al., 2014; Falcone et al., 2016) and p40^phox^-deficient mice were more susceptible to DSS colitis than wild-type mice (Conway et al., 2012). One explanation for these differences may be individual roles of each subunit in NOX-independent signaling pathways. On the other hand, external environmental influences such as the prevalence of commensal/pathogenic microorganisms may contribute to the variability, particularly as the microbiota has a large impact on IBD (Nell et al., 2010; Perše and Cerar, 2012). Finally, the mechanism of colitis induction is probably critical. Recently, a study demonstrated that mice with a hypomorphic mutation in *Cyba* (p22^phox^) showed loss of the mucus layer, dysbiosis, and increased inflammation while *Cyba*-deficient mice did not display any predisposition to DSS colitis (Aviello et al., 2019). Notably, ROS generation in neutrophils was also absent in the mice with the hypomorphic mutation, but, opposed to the complete p22^phox^ deficiency, NOX4 remained functional. Hence, compensation by other ROS sources in the intestine, e.g., NOX4 in epithelial cells, may affect the disease phenotype, at least in rodents.

## Conclusion

Intensive studies in human and mouse systems have led to a comprehensive understanding of the contribution of phagocyte-derived ROS to health and disease. Yet, gaps of knowledge remain especially with regard to the specific targeting of individual ROS sources or the transferability of results originating in rodent models. As one example, NOX2-deficient mice do not spontaneously develop intestinal bowel disease, which is a prevalent symptom of CGD patients. On the other hand, the conservation of the signaling components in ROS pathways presents also an opportunity for performing studies in animals of lower complexity. *Drosophila* might be an excellent model to study the effects of mitochondrial ROS (Salminen and Vale, 2020), considering the availability of suitable genetic tools. The zebrafish, on the other hand, exhibits a CGD-like phenotype upon NOX2 deficiency (Schoen et al., 2020) and offers the possibility to investigate the individual role of ROS in both granulocytes and mononuclear phagocytes.

A more profound knowledge of the involved pathways and downstream effects is crucial, as both an excessive and a diminished production of ROS have proven to be harmful. Additionally, the development of specific inhibitors, e.g., small molecules or plant-based substances, is still in its infancy (Panday et al., 2015). Further research in this area will thus serve the purpose of not only developing more specific therapeutics for CGD, for which the current standard therapy is bone marrow transplantation, but also understanding the regulation of a balanced immune response in general.

## Author Contributions

ZM, PH, and JK wrote and edited the manuscript. All authors contributed to the article and approved the submitted version.

## Conflict of Interest

The authors declare that the research was conducted in the absence of any commercial or financial relationships that could be construed as a potential conflict of interest.
